# A Study on Trauma Mechanisms and Injury Sites in Patients with Blunt Abdominal Trauma

**DOI:** 10.1155/2022/2160766

**Published:** 2022-07-13

**Authors:** YoungUn Choi, SuHyun Kim, JiWool Ko, MyoungJun Kim, Hongjin Shim, JaeHun Han, JiHye Lim, Kwangmin Kim

**Affiliations:** ^1^Department of Surgery, Yonsei University Wonju College of Medicine, Wonju 26426, Republic of Korea; ^2^Trauma Center, Wonju Severance Christian Hospital, Wonju 26426, Republic of Korea; ^3^Wonju Severance Trauma Research Group, Yonsei University Wonju College of Medicine, Wonju 26426, Republic of Korea; ^4^National Health Big Data Clinical Research Institute, Yonsei University Wonju College of Medicine, Wonju 26426, Republic of Korea

## Abstract

**Background:**

Although blunt abdominal trauma is sometimes readily identified in patients with trauma, its diagnosis and treatment can be delayed due to various limitations including unconsciousness or unstable vital functions, which may cause shock due to blood loss and sepsis. Confirming the correlation between the specific damage of the abdominal organ and the recommended surgical intervention will allow for predicting abdominal damage based on the specific underlying trauma mechanisms.

**Objectives:**

This study aimed to assess the proportion of patients with blunt trauma resulting from intraabdominal injury who received surgical intervention (surgery and angioembolization [A/E]), stratified by trauma mechanism and to examine which organs were damaged per different trauma incident.

**Methods:**

We retrospectively analyzed the clinical characteristics of 2,291 patients in a tertiary trauma center. Clinical characteristics included age, sex, injury severity score, trauma mechanism (car, motorcycle, pedestrian, bicycle, ship or train accident, fall, slipping or rolling down, bumping, crush injury, explosion burn, and others), abdominal surgical intervention, damaged organ, and A/E site.

**Results:**

One-fourth of the patients with blunt trauma required surgical intervention in the abdomen. In particular, the mesentery or bowel was the main injured area for abdominal surgery in all mechanisms, and the spleen or liver was the main damaged organ subjected to A/E. Therefore, we should consider that a substantial proportion of patients with trauma do require abdominal surgery. In particular, repeated physical examination and imaging tests are necessary when the patients are unconscious or their vital functions are unstable for accurate confirmation of injury.

## 1. Introduction

According to the Statistical Yearbook of the Trauma Registration System of the National Emergency Medical Center, the number of visits of patients with trauma from 17 medical institutions selected as regional trauma centers in Korea was 34,318 in 2020 [1]. Most of them were due to blunt trauma accidents, and the percentage of traffic accidents was the highest (33.8%) followed by slipping, falling, and crushing. In addition, the patients with polytrauma constituted 48.4% of all patients with trauma, but 81.1% of patients with trauma bore an injury severity score (ISS) of 16 or higher. Abdominal damage was confirmed in 19.4% of all patients with trauma and in 37.3% of patients with severe trauma, but which specific abdominal organs were damaged by which trauma mechanism and at what rate surgical intervention was performed were not investigated. Research on these remain scarce. In particular, it is difficult to trust the physical examination of the abdomen during initial assessments in unconscious patients with head injury [2–5]. In addition, very small amounts of fluid accumulated in the abdominal cavity due to bowel perforation or mesenteric injury from blunt injury can easily be missed using imaging tools such as focused assessment with sonography in trauma (FAST) or computed tomography (CT) [6, 7], and in such unstable cases, it is also difficult to proceed with CT. Damage in several areas due to polytrauma and unstable vital functions can also cause difficulty in CT assessment. The purpose of this study was to determine the proportion of patients with blunt trauma who received surgical treatment (surgery and angioembolization [A/E]) due to intraabdominal injury in each trauma mechanism and to identify which intraabdominal organ was damaged. If the relationship between specific organ damage and surgery according to a specific mechanism is established, it will be possible to predict abdominal damage according to the specific mechanisms implicated in trauma.

## 2. Materials and Methods

We retrospectively reviewed the data of patients with trauma transferred to the emergency room from March 1, 2015, to August 31, 2021, excluding patients transferred from other hospitals after completing acute treatment, patients deceased upon arrival, pregnant women, patients with no medical records, or patients who objected to treatment. Age, sex, ISS score, trauma mechanisms, and abdominal surgical intervention (surgery or A/E) were analyzed in 2,291 patients. The trauma mechanisms were divided into car accident, motorcycle accident, pedestrian accident, bicycle accident, ship or train accident, fall, slipping and rolling down, bumping injury, crush injury, explosion burn, and others, and abdominal injury sites were divided into liver, spleen, bowel, mesentery and omentum, pancreas, kidney, bladder, and others. In the case of A/E, target organs were classified into the liver, spleen, pelvis, and others. Using this data, the frequency and order of abdominal surgery sites and the angiography sites for each mechanism were checked. This study was approved by the our institutional review board (IRB No. CR 321156).

## 3. Statistical Analysis

Data were expressed as the mean ± standard deviation for continuous variables and frequency (percentages) for categorical variables. The chi-squared test was used for categorical variable analysis. One sample proportion test was performed to test the difference in proportion. All statistical analyses were performed using SAS version 9.4 (SAS Institute, Cary, North Carolina, US) and R version 3.6.3 (R core Team, Vienna, Austria). Statistical significance was set to *P*=0.05.

## 4. Results

Of the 2,291 patients, 1,605 (70.1%) were men, and the most common trauma mechanisms were car accident (42.08%), falls (23.26%), pedestrian accidents (11.31%), and motorcycle accidents (9.04%) (Table 1, Figure 1). There was no significant difference in ISS score and average age for each of these mechanisms. Five hundred sixty-two patients (24.53%) received surgical intervention for abdominal injury, and 399 (17.4%) received abdominal surgery (Figure 2). Among them, the ratio of the mesentery and bowel was the highest at 54.14% and 37.59%, respectively (Table 1, Figure 3). A/E was performed in 163 patients (7.1%) (Figure 2), and the ratio of the spleen and liver was the highest at 46.01 and 31.29% (Table 1, Figure 4). In all mechanisms, the rate of abdominal surgery was highest for car accidents with 224 cases (23.2%) and mesentery and bowel being the most frequent sites, and A/E was the highest in pedestrian accidents with 35 cases (13.5%) and the spleen, pelvis, and liver being the most frequent sites.

For mechanisms with more than 20 patients, abdominal surgery and A/E were performed with almost the same frequency in mechanisms C (pedestrian accident) and D (bicycle accident) (Table 2).

For each mechanism, a ratio test was performed on a site with high frequency in relation to the surgical and A/E sites. Here, if the sample size is too small, the test is meaningless, so the test was not performed on surgical mechanisms with a sample number of less than 10. In the case of surgery, the ratio of mesentery and bowel surgery was high for most of the mechanisms, and it was confirmed that the operation was performed in the order of the mesentery > bowel > liver with statistical significance in specific car and pedestrian accidents. In the case of A/E, the ratio of the spleen and liver was confirmed to be overall high, and in car accidents, we confirmed that the progression was statistically significant and followed the order of the spleen > liver > pelvis (Table 3).

Since traffic accidents accounted for most trauma cases, the mechanisms were compared separately for traffic accidents and nontraffic accidents. In both groups, it was confirmed that the operation was performed in the order of the mesentery > bowel > liver, and A/E was performed in the order of the spleen > liver > pelvis (Table 4). Since the *P* value is higher than 0.005, we confirmed that surgery and A/E are proceeding in the same sequence without any difference between the two groups.

## 5. Discussion

Organ damage caused by a blunt abdominal injury is mainly caused by deceleration, external compression, and crushing injury [8]. Deceleration creates a shearing force that causes the immobilized organ to be torn. In addition, if pressure is suddenly applied to the abdomen from the outside and the intraabdominal pressure rises, the intestine may be ruptured, and the abdominal organs may be compressed and damaged due to the high pressure acting between the abdominal wall and the spine [9]. A blunt abdominal injury can damage the spleen, liver, intestine, mesentery, and pancreas.

Clinical symptoms appear in various forms such as abdominal stiffness and distension, tenesmus, and nausea or be asymptomatic. Methods such as sonography and CT including P/E are used for diagnosis during initial assessment of patients with trauma. Unfortunately, in the severely injured patients, polytrauma and head and neck injuries are very common (68.1%) [1]. Accordingly, to trust the abdominal P/E of unconscious patients during the initial assessment can be difficult. In addition, in the case of polytrauma in which the patient's life is threatened, including bleeding from multiple sources, it is difficult to proceed with CT in the initial stage. Moreover, even if CT is performed, if the transfer time from the site of injury to the emergency room (ER) is not long, intraabdominal fluid collection due to bowel injury or organ damage is small and may not be clearly confirmed by imaging [10, 11]. Even a rupture of the abdominal diaphragm may not be confirmed by CT. In such situations, sepsis may occur due to peritonitis and massive intraabdominal hemorrhage. In addition, the presence of ascites, liver cirrhosis, or chronic renal failure with peritoneal dialysis can mask the intraabdominal bleeding of patients with trauma.

In general, patients with solid organ and severe pelvic injury accompanied by active bleeding can be treated using A/E [12, 13]. Laparotomy is actively recommended when bowel injury is suspected, the patient is hemodynamically unstable, and intraabdominal bleeding is confirmed [14]. In this study, we verified that one-fourth of patients with trauma underwent surgical intervention for abdominal injury, and the proportion of the latter was similar to that of patients with trauma in Korea in 2020. We also confirmed that the mesentery and bowel accounted for 91.73% of the cases of abdominal surgery. Therefore, when the P/E is unreliable because the patient bearing the trauma is unconscious or when the abdominal CT scan is limited due to unstable vitality, we must always consider the possibility of intraabdominal injury and reduce possible misdiagnosis through repeated P/E and FAST.

## 6. Limitations

This study bears certain limitations. First, the treatment for patients diagnosed with blunt abdominal trauma involved observation, laparotomy, and A/E. Even when intraabdominal injuries were diagnosed at the time of injury, the observation groups were not included in the surgical intervention in this study. In such cases, conservative treatment was performed, such as for grade 1 and 2 liver injury and spleen laceration. Second, for pelvic injury, preperitoneal pelvic packing (PPP) was not included in laparotomies. Regarding patients with severe pelvic bone injury, in whom A/E and PPP should be done first, there may exist differences in policy for each institution, the surgeon's experience and opinion, and the availability of the radiologist. However, in this study, PPP was not considered an intraperitoneal operation and was included in the A/E site. Third, trauma cases that were not treated by the trauma team due to being referred to the acute care surgery team were possibly excluded from follow-up. Therefore, it is possible that some trauma cases were omitted from the record. Fourth, patients who were transferred after completing acute treatment at other hospitals and patients who had undergone surgical treatment for abdominal injuries may have been excluded as well. Fifth, even with the same trauma mechanism, the accident cause may vary; therefore, it is not certain that a specific mechanism will clearly represent a specific injury cause. For example, in the case of a pedestrian accident, the abdominal cavity damage area will be different depending on which part of the body collides with which type of the vehicle in which direction. Therefore, a specific mechanism may cause damage to different body areas.

## 7. Conclusions

One-fourth of blunt patients with trauma transferred to the ER required surgical intervention (surgery or A/E) for abdominal injury, and surgery was performed with the frequency order of the mesentery > bowel > liver. Abdominal injury was confirmed to be significant in car and pedestrian accidents. A/E was performed in the order of frequency of the spleen > liver > pelvis and was significantly confirmed for car accidents. When the traffic accident group which is the most common cause and the nontraffic accident group were divided and compared, there was no difference in the specific abdominal injury site that received surgical intervention. Therefore, the mesentery and bowel are the main injured areas requiring abdominal surgery in all injury mechanisms, and the spleen and liver are the main damaged organs that require to be subjected to A/E.

When assessing patients with trauma, we need to consider that one-fourth of them will bear an abdominal injury that requires surgical intervention. In particular, accurate confirmation of repeated P/E and imaging tests is necessary, especially when the patient is unconscious or their vital functions are unstable.

## Figures and Tables

**Figure 1:** The percentage of patients that experienced each type of trauma mechanism.

**Figure 2:** Ratio of surgery and angioembolization by each trauma mechanism. A, car accident; B, motorcycle accident; C, pedestrian accident; D, bicycle accident; E, ship or train accident; F, fall; G, slipping and rolling down; H, bumping injury; I, crush injury; J, explosion burn; K, others; 1, liver; 2, spleen; 3, bowel; 4, mesentery and omentum; 5, pancreas; 6, kidney; 7, bladder; 8, others.

**Figure 3:** Proportion of abdominal surgery sites by trauma mechanisms. A, car accident; B, motorcycle accident; C, pedestrian accident; D, bicycle accident; E, ship or train accident; F, fall; G, slipping and rolling down; H, bumping injury; I, crush injury; J, explosion burn; K, others; 1, liver; 2, spleen; 3, bowel; 4, mesentery and omentum; 5, pancreas; 6, kidney; 7, bladder; 8, others.

**Figure 4:** Proportion of abdominal angiography sites by trauma mechanisms. A, car accident; B, motorcycle accident; C, pedestrian accident; D, bicycle accident; E, ship or train accident; F, fall; G, slipping and rolling down; H, bumping injury; I, crush injury; J, explosion burn; K, others; 1, liver; 2, spleen; 3, pelvis; 4, others.

**Table 1:** Patients' clinical characteristics and frequency of surgery and angiography according to each trauma mechanism.

Variables	Overall	A	B	C	D	E	F	G	H	I	J	K
	*N*= 2,291	*N*= 964	*N*= 207	*N*= 259	*N*= 48	*N*= 53	*N*= 533	*N*= 51	*N*= 146	*N*= 16	*N*= 4	*N*= 10
Age	49.4 ± 19.0	48.5 ± 17.4	43.8 ± 22.0	52.4 ± 22.1	43.4 ± 26.1	65.3 ± 15.0	49.6 ± 17.8	51.7 ± 23.5	51.5 ± 16.5	59.5 ± 9.4	42.0 ± 16.8	49.5 ± 17.3

Sex												
Female patients	686 (29.9)	375 (38.9)	22 (10.6)	102 (39.4)	9 (18.8)	8 (15.1)	124 (23.3)	21 (41.2)	23 (15.8)	1 (6.3)	0 (0.0)	1 (10.0)
Male patients	1605 (70.1)	589 (61.1)	185 (89.4)	157 (60.6)	39 (81.3)	45 (84.9)	409 (76.7)	30 (58.8)	123 (84.3)	15 (93.8)	4 (100)	9 (90.0)

ISS	16.4 ± 10.7	13.7 ± 9.9	17.6 ± 10.6	21.1 ± 11.8	19.4 ± 14.2	15.7 ± 8.6	18.6 ± 10.4	12.8 ± 7.6	15.1 ± 7.8	23.1 ± 18.5	30.3 ± 20.4	19.6 ± 10.1

Surgery												
No	1892 (82.6)	740 (76.8)	166 (80.2)	222 (85.7)	43 (89.6)	40 (75.5)	495 (92.9)	45 (88.2)	119 (81.5)	10 (62.5)	4 (100)	8 (80.0)
Yes	399 (17.4)	224 (23.2)	41 (19.8)	37 (14.3)	5 (10.4)	13 (24.5)	38 (7.1)	6 (11.8)	27 (18.5)	6 (37.5)	0 (0.0)	2 (20.0)
1	66 (2.9)	29 (3.0)	9 (4.3)	7 (2.7)	2 (4.2)	2 (3.8)	13 (2.4)	0 (0.0)	2 (1.4)	1 (6.3)	0 (0.0)	1 (10.0)
2	56 (2.4)	21 (2.2)	10 (4.8)	5 (1.9)	1 (2.1)	3 (5.7)	9 (1.7)	2 (3.9)	5 (3.4)	0 (0.0)	0 (0.0)	0 (0.0)
3	150 (6.5)	96 (10.0)	12 (5.8)	9 (3.5)	0 (0.0)	5 (9.4)	12 (2.3)	1 (2.0)	9 (6.2)	5 (31.3)	0 (0.0)	1 (10.0)
4	216 (9.4)	138 (14.3)	17 (8.2)	16 (6.2)	1 (2.1)	7 (13.2)	17 (3.2)	2 (3.9)	11 (7.5)	6 (37.5)	0 (0.0)	1 (10.0)
5	19 (0.8)	10 (1.0)	4 (1.9)	2 (0.8)	0 (0.0)	1 (1.9)	2 (0.4)	0 (0.0)	0 (0.0)	0 (0.0)	0 (0.0)	0 (0.0)
6	14 (0.6)	4 (0.4)	4 (1.9)	2 (0.8)	0 (0.0)	0 (0.0)	2 (0.4)	0 (0.0)	1 (0.7)	0 (0.0)	0 (0.0)	1 (10.0)
7	15 (0.7)	3 (0.3)	1 (0.5)	5 (1.9)	1 (2.1)	0 (0.0)	2 (0.4)	1 (2.0)	1 (0.7)	0 (0.0)	0 (0.0)	1 (10.0)
8	21 (0.9)	10 (1.0)	0 (0.0)	7 (2.7)	0 (0.0)	1 (1.9)	1 (0.2)	0 (0.0)	2 (1.4)	0 (0.0)	0 (0.0)	0 (0.0)

Angiography												
No	2128 (92.9)	909 (94.3)	190 (91.8)	224 (86.5)	44 (91.7)	50 (94.3)	506 (94.9)	47 (92.2)	133 (91.1)	14 (87.5)	3 (75.0)	8 (80.0)
Yes	163 (7.1)	55 (5.7)	17 (8.2)	35 (13.5)	4 (8.3)	3 (5.7)	27 (5.1)	4 (7.8)	13 (8.9)	2 (12.5)	1 (25.0)	2 (20.0)
9	51 (2.2)	18 (1.9)	8 (3.9)	10 (3.9)	2 (4.2)	0 (0.0)	6 (1.1)	1 (2.0)	2 (1.4)	2 (12.5)	1 (25.0)	1 (10.0)
10	75 (3.3)	34 (3.5)	6 (2.9)	13 (5.0)	1 (2.1)	1 (1.9)	10 (1.9)	3 (5.9)	6 (4.1)	0 (0.0)	0 (0.0)	1 (10.0)
11	36 (1.6)	6 (0.6)	3 (1.4)	13 (5.0)	1 (2.1)	1 (1.9)	10 (1.9)	0 (0.0)	2 (1.4)	0 (0.0)	0 (0.0)	0 (0.0)
12	16 (0.7)	5 (0.5)	1 (0.5)	1 (0.4)	0 (0.0)	1 (1.9)	3 (0.6)	0 (0.0)	4 (2.7)	1 (6.3)	0 (0.0)	0 (0.0)

A, car accident; B, motorcycle accident; C, pedestrian accident; D, bicycle accident; E, ship or train accident; F, fall; G, slipping and rolling down; H, bumping injury; I, crush injury; J, explosion burn; K, others; 1, liver; 2, spleen; 3, bowel; 4, mesentery and omentum; 5, pancreas; 6, kidney; 7, bladder; 8, others; 9, liver; 10, spleen; 11, pelvis; 12, others; ISS, injury severity score. Data are expressed as *n* (%) or the mean (±standard deviation) unless otherwise specified.

**Table 2:** Frequency of surgery and angiography according to trauma mechanisms.

		Overall	A	B	C	D	E	F	G	H	I	J	K
		*N*= 2,291	*N*= 964	*N*= 207	*N*= 259	*N*= 48	*N*= 53	*N*= 533	*N*= 51	*N*= 146	*N*= 16	*N*= 4	*N*= 10
Surgery	Angiography												

No	No	1747 (76.3)	694 (72.0)	150 (72.5)	192 (74.1)	39 (81.3)	37 (69.8)	470 (88.2)	41 (80.4)	107 (73.3)	8 (50.0)	3 (75.0)	6 (60.0)
	Yes	145 (6.3)	46 (4.8)	16 (7.7)	30 (11.6)	4 (8.3)	3 (5.7)	25 (4.7)	4 (7.8)	12 (8.2)	2 (12.5)	1 (25.0)	2 (20.0)

Yes	No	381 (16.6)	215 (22.3)	40 (19.3)	32 (12.4)	5 (10.4)	13 (24.5)	36 (6.8)	6 (11.8)	26 (17.8)	6 (37.5)	0 (0.0)	2 (20.0)
	Yes	18 (0.8)	9 (0.9)	1 (0.5)	5 (1.9)	0 (0.0)	0 (0.0)	2 (0.4)	0 (0.0)	1 (0.7)	0 (0.0)	0 (0.0)	0 (0.0)

A, car accident; B, motorcycle accident; C, pedestrian accident; D, bicycle accident; E, ship or train accident; F, fall; G, slipping and rolling down; H, bumping injury; I, crush injury; J, explosion burn; K, others. Data are expressed as *n* (%).

**Table 3:** Ranking of abdominal surgery and angiography site frequency by trauma mechanism.

Variables	Mechanism										
	A	B	C	D	E	F	G	H	I	J	K
Injury site (surgery)											
ranking	4 > 3> 1	4 > 3> 2	4 > 3> 1 = 8	1 > 2 = 4 = 7	4 > 3> 2	4 > 1> 3	2 = 4 > 3 = 7	4 > 3> 2	4 > 3> 1	—	1 = 3 = 4 = 6 = 7
*P* value	**<0.001**	0.0704	**0.009**	—	0.207	0.1179	—	0.275	0.394	—	—

Injury site (angiography)											
ranking	10 > 9> 11	9 > 10> 11	10 = 11 > 9	9 > 10 = 11	10 = 11 = 12 > 9	10 = 11 > 9	10 > 9 > 11 = 12	10 > 12 > 9 = 11	9 > 12 > 10 = 11	9 > 10 = 11 = 12	9 = 10 > 11 = 12
*P* value	**<0.001**	0.2171	0.1763	—	—	0.0600	—	0.1982	—	—	—

A, car accident; B, motorcycle accident; C, pedestrian accident; D, bicycle accident; E, ship or train accident; F, fall; G, slipping and rolling down; H, bumping injury; I, crush injury; J, explosion burn; K, others; 1, liver; 2, spleen; 3, bowel; 4, mesentery and omentum; 5, pancreas; 6, kidney; 7, bladder; 8, others; 9, liver; 10, spleen; 11, pelvis; 12, others. *P* value was calculated by proportion test.

**Table 4:** Correlation between the traffic accident and the abdominal surgery site.

Variables	Traffic collisions		
	No	Yes	*P*-value
Injury site (surgery)			0.2540
1	17 (15.2)	49 (11.0)	
2	16 (14.3)	40 (9.0)	
3	28 (25.0)	122 (27.4)	
4	37 (33.0)	179 (40.2)	
5	2 (1.8)	17 (3.8)	
6	4 (3.6)	10 (2.3)	
7	5 (4.5)	10 (2.3)	
8	3 (2.7)	18 (4.0)	
Ranking	**4** **>** **3>** **1**	**4** **>** **3>** **1**	
*P*-value	**0.032**	**<0.001**	

Injury site (angiography)			0.2465
9	13 (24.5)	38 (30.4)	
10	20 (37.7)	55 (44.0)	
11	12 (22.6)	24 (19.2)	
12	8 (15.1)	8 (6.4)	
Ranking	**2** **>** **1>** **3**	**2** **>** **1>** **3**	
*P*-value	**0.024**	**<0.001**	

1, liver; 2, spleen; 3, bowel; 4, mesentery and omentum; 5, pancreas; 6, kidney; 7, bladder; 8, others; 9, liver; 10, spleen; 11, pelvis; 12, others. *P* value was calculated by the proportion test.

## Data Availability

The datasets used during and/or analyzed during the current study are available from the corresponding author on reasonable request.
